The article "Recognizing Decision-Making Using Eye Movement: A Case Study With Children" was published in 2020. Journal: Front Psychol.

# Recognizing Decision-Making Using Eye Movement: A Case Study With Children

**DOI:** 10.3389/fpsyg.2020.570470

**Published:** 2020-09-24

**Authors:** Juan-Carlos Rojas, Javier Marín-Morales, Jose Manuel Ausín Azofra, Manuel Contero

**Affiliations:** ^1^Escuela de Arquitectura, Arte y Diseño, Tecnologico de Monterrey, Monterrey, Mexico; ^2^I3B – Instituto de Investigación e Innovación en Bioingeniería, Universitat Politècnica de València, Valencia, Spain

**Keywords:** eye movements, recognizing, decision-making, children, product

## Abstract

The use of visual attention for evaluating consumer behavior has become a relevant field in recent years, allowing researchers to understand the decision-making processes beyond classical self-reports. In our research, we focused on using eye-tracking as a method to understand consumer preferences in children. Twenty-eight subjects with ages between 7 and 12 years participated in the experiment. Participants were involved in two consecutive phases. The initial phase consisted of the visualization of a set of stimuli for decision-making in an eight-position layout called Alternative Forced-choice. Then the subjects were asked to freely analyze the set of stimuli, they needed to choose the best in terms of preference. The sample was randomly divided into two groups balanced by gender. One group visualized a set of icons and the other a set of toys. The final phase was an independent assessment of each stimulus viewed in the initial phase in terms of liking/disliking using a 7-point Likert scale. Sixty-four stimuli were designed for each of the groups. The visual attention was measured using a non-obstructive eye-tracking device. The results revealed two novel insights. Firstly, the time of fixation during the last four visits to each stimulus before the decision-making instant allows us to recognize the icon or toy chosen from the eight alternatives with a 71.2 and 67.2% of accuracy, respectively. The result supports the use of visual attention measurements as an implicit tool to analyze decision-making and preferences in children. Secondly, eye movement and the choice of liking/disliking choice are influenced by stimuli design dimensions. The icon observation results revealed how gender samples have different fixation and different visit times which depend on stimuli design dimension. The toy observations results revealed how the materials determinate the largest amount fixations, also, the visit times were differentiated by gender. This research presents a relevant empirical data to understand the decision-making phenomenon by analyzing eye movement behavior. The presented method can be applied to recognize the choice likelihood between several alternatives. Finally, children’s opinions represent an extra difficulty judgment to be determined, and the eye-tracking technique seen as an implicit measure to tackle it.

## Introduction

The novel collaboration between consumer, scientist, and marketing experts leads to better identification, recognition, and understanding of consumer behavior. Self-report and behavioral measurements are the instruments that have been used to study the consumer’s experience, thoughts, and emotions. In the last decade, the use of self-report surveys and visual representation tools has demonstrated how people can describe their reactions and decision-making process in choosing products and services (Poels and Dewitte, 2006). Advances in neurosciences, neurobiology, and neuropsychology increase our knowledge of how brain works (Crone and Ridderinkhof, 2011; Blanco et al., 2014), and how reality is interpreted through daily-life experiences, the interaction with the environment, and daily decision-making (Lăzăroiu, 2017).

The contributions generated by applying concepts of neuroscience to consumer research have been significant due to the application of physiological measures in the last years (Hubert and Kenning, 2008; Wang and Minor, 2008; Solnais et al., 2013; Hubert, 2010). Karmarkar and Plassmann (2017) discuss extensively the integration of neurophysiological data in consumer research, mainly describing the ability of consumer behavior prediction and decision-making, breaking boundaries established by conventional techniques. Neuroscience techniques offer the ability to recognize implicit measurements not controlled by conscious processes (Lieberman, 2007), revealing cognitive process that can be approached from the modifications of sensory stimuli to people’s attention elements (Ochsner and Gross, 2005). Advances in the application of implicit measurements have led to a wide range of physiological measurement techniques to be now considered as tools for consumer recognition. These tools are considered a step ahead in self-report in consumer research (Bell et al., 2018), which should be reviewed for deeper application. Some of the most used tools for physiological measurement are electroencephalogram (EEG), functional MRI (fMRI), electrodermal activity (EDA), heart rate (HR), and eye movement (also, eye-tracking; Wedel and Pieters, 2006; Smidts et al., 2014; Hsu and Yoon, 2015; Hsu, 2017; Karmarkar and Plassmann, 2017; Bell et al., 2018).

Eye movement or gaze attention is a widely used tool to assess people’s behavior, including children, in order to know which visual stimuli are liked and chosen. Mitsura and Glaholt (2014) demonstrated how gaze behaves more strongly in a liking decision than dislike decision, and also the young participants in the study were not greatly influenced by the categorization of the stimuli. The relationship between eye-movements and preference has been studied repeatedly, but research with samples of children is limited. Old studies of eye movement have demonstrated its application to identify preferences, even in children. They show that if a stimulus is observed more times, that is the preferred one (Fantz, 1963, 1964). Measuring gaze and how it affects decision-making provides important information on the nature of stimuli, and attention level can stimulate the consumer preference (Djamasbi, et al., 2010; Rojas et al., 2015; Van der Laan et al., 2015; Yaramothu et al., 2018; Qu and Gou, 2019; Steinhauser et al., 2019). Shimojo et al. (2003) and Simion and Shimojo (2006, 2007) explained the first indicator of a gaze bias that exists during selection between two visually present stimuli. The experimentation with two elements presented and selected on attractiveness showed that eye movement is biased toward the element that was later selected. This gaze bias becomes evident between 1 and 1.5 s prior to the response that marked the overt decision. Other studies have shown that the observed stimulus is an important factor for generating an attentive gaze (Park et al., 2010; Liao et al., 2011). One of these studies replicates a two-alternative preference judgment task between a new stimulus and a repeatedly know stimulus. The results indicated that a facial stimulus is more familiar than any other type of stimulus. Recently, Morii and Sakagami (2015) showed how the gaze cascade effect phenomenon is an indicator of preferred judgment, where the choice of a stimulus is within the viewing time. However, the selection between two alternatives often does not correspond to the reality of decision-making between stimuli. Glaholt et al. (2009) demonstrated that the bias in looking behavior was particularly robust in eight-alternative forced-choice (8-AFC) decision tasks. These findings imply that, by monitoring eye movements, it may be possible to recognize the observers’ selection or preference prior to the overt response and possibly prior to the point at which the selection is consciously made. In another experiment, Glaholt and Reingold (2012) replicated the effect of modulating visual attention and decision-making of a stimulus observed in an arrangement of several images, obtaining similar results.

The potential of the eye movement method can reveal information about children’s gaze behavior. In contrast, according to the literature related to self-reports, children can be assessed through different traditional methods, but there are multiple limitations such as age-group of interest, styling of self-report instruments, response formats for self-report, language, space contamination, concrete or styling stimuli, and design elements to consider (Song et al., 1994; Chambers, 2002; Sturgess et al., 2002; Kuijpers et al., 2014). This limitation types gives partial information when we use self-report, however, possibilities using the implicit measure combined the traditional assessment and gaze or eye movement can support a novel consumer research. In the same line of thought, the gaze can provide a predictive application for choice alternatives. Previous findings have shown the contribution to consumer behavior understanding through an implicit measure, and implication in decision-making process through the gaze. In order to measure the children’s attention in Saegusa et al. (2015) experiment, stimuli were designed such these could be attractive and familiar to the sample. In similar experiments, there is a justification for understanding the attractiveness of certain stimuli to people.

Another reasoning for the choice of recognizable or familiar stimuli is the heuristic recognition theory and the research on the processing of decision-making according to a few researches of the last years. Marewski et al. (2009) suggest that simple cognitive mechanisms may outperform complex cognitive processes that are mostly noise in people’s minds. Simple judgments should not require complex understanding. Furthermore, Arkes et al. (2016) argue that consistency is a basic rule to understand behavior. So too, coherence plays a key role in situations where it is instrumental in achieving functional goals. In the last decade, Gigerenzer and Goldstein (2011) have described how judgment and decision-making can be described as a simple heuristic model. Also, Pachur et al. (2011) opened the debate on the processes underlying the use of recognition in decision-making. The authors suggest that recognition is often an ecologically valid signal, that people often follow recognition when making inferences. In terms of human behavior, recognition seems to have a special status in decision-making.

For this research, we include elements that are familiar and that will be easily recognized by the participants. For example, faces are a stimulus that has a level of attractiveness or beauty that is often associated with desire. In addition, faces are associated with emotional aspects (Saegusa et al., 2015) and the familiarity that these can represent to a person to leads to preference (Liao et al., 2013) and recognize the capacity of remind aspect related to consumer experience (Heljakka and Ihamäki, 2019). The stimulus, due to its familiarity, can change a consumer’s decision-making process. The visual attention that a familiar stimulus can represent can be full of emotional components and attractive physical attributes. There is an enormous relationship between good physical attributes with good emotional components in product configuration (Hertenstein et al., 2013), and the attractiveness generated by this (Joško-Brakus et al., 2014; Kareklas et al., 2014), transmitted through different visual media (physical or digital), can affect decision-making or preference (Cowart et al., 2008; Cho and Kim, 2012).

Tanaka et al. (2001) distinguished three basic attributes to perceive objects: shape, color, and texture. These three attributes give a complete “object representation” leading to more complex cognitive processes, giving us the ability to understand the visual elements. Through form, texture, objects, color, and intensities, a familiar stimulus to children could stand out and serve as an attraction to attractor the consumer’s attention (Kwon et al., 2002; Luo, 2006; Lin, 2010; Festila and Chrysochou, 2018). Specifically, color plays a fundamental role as a factor of aesthetic attractiveness to everybody, from a perceptual aspect (Helo et al., 2014) to the emotional aspect (Green-Armytage, 2006). Various studies have demonstrated the importance and influence of such attributes (related with brands) on the perceived quality of a product (Grunert et al., 2004; Laforet, 2011). In our case configuration, the stimuli are provided by toys to manage and facilitate their visualization by and familiarization with children, just as in the examples described by Hult et al. (2019) for consumer experience.

The aim of this paper is to examine, through stimuli designed with elements familiar to children, attractive attributes and emotional components, the decision-making recognition when showing different stimuli alternatives in 8-AFC decision tasks and traditional assessment of the stimuli. The implementation of an implicit measure will support the limitation, difficulty, and even the ethical implications of using children as a sample for this research or any type of sample in similar studies (Stanton et al., 2017). The information that this investigation will give us using the behavior of gaze as an implicit measure can contribute to the comparison of physiological measures and self-reports.

## Materials and Methods

### Participants

This study was conducted with 30 children aged 7–12 years, divided in two groups for the two groups of stimuli. Twenty-eight children (14 girls, *M* = 9.5 years; *SD* = 1.7) took part in the experiment. The parents’ permission was requested to conduct the experiments. All methods and experimental protocols were performed in accordance with the guidelines and regulations of the local ethics committee of the Polytechnic University of Valencia.

### Instrumentation

An unobtrusive eye tracker capable of recording the position of the eyes at a sampling rate of 300 Hz (Tobii TX300, Tobii, Stockholm, Sweden) was used to measure the participants’ visual fixations. This device has a 23″ flat HD screen and a sensor bar in the lower part of it. This setup allows participants to make large head movements, and to move freely and naturally in front of the screen. Tobii Studio 3.2.1 software was used to calibrate the eye tracker, to present the stimuli and record the data.

### Stimuli

For the experiment, two groups of stimuli were created following a simple design base. Icons and toys were designed and constructed with a unique combination of three stimulus dimensions. The first group (icon) used as dimensions: a character (animal), a color, and a detail eye. For each dimension, five options were selected to create 125-possible combination of icons. The second group (toys) was designed follow the same construction, three dimensions were used: a character (animal), a color, and a material. For each dimension, five options were selected to create 125-possible combination of toys. However, the 125 combinations for each group were not used due to the length of the study, thus it was decided to only take 64 randomly selected combinations from the original set for the experiment. All the possible combinations are shown in Figure 1. We verified that the frequency of occurrence the five elements of the icon and toy design had a uniform distribution.

**Figure 1:** Stimuli dimensions for icons and toys design.

### Procedure

The experiment consisted of two tasks that were completed by the participants in a fixed order: 8-AFC and individual visual and verbal evaluation. The sample was randomly divided into two groups balanced by gender. One group of participants was given the icons version of the experiment, and other group was given the toys version. Each participant was given instructions before participating in each component of the experiment. A preparation task was designed to instruct on the 8-AFC task to be performed by the young participants. A complete scheme of the task can be seen in Figure 2.

**Figure 2:** Complete scheme of the task in the experiment.

The first task included the tracking measurement using the method 8-AFC (Glaholt and Reingold, 2009, 2012; Mitsura and Glaholt, 2014) in terms of choice likelihood, in a layout of 3 × 3 boxes, which serves to distribute the eight different options of the 64 icons or toys selected. The stimuli were spread in every box except the central box; inside of this box, a black point is displayed as an indicator to complete task. To begin, the participant had to freely watch the eight different options and choose the favorite one with no limit of time. After that, when the subjects know what stimuli will be chosen, the gaze must move to the black point just for 2 s. Then, the black point turns green color, indicating the beginning of the decision-making part of the task. The participant must return to watch the favorite stimuli to indicate their liking choice using gaze feedback (see Figure 3). Eight layouts were designed to cover the 64 combinations of icons and toys. The second task was to perform an independent assessment of each stimuli using a Likert-scale. The same 64 icons and toys from the first task were taken to create a layout for every stimulus. With every stimulus, a Likert-scale (1, I do not like and 7, I like it) was included and the participant made a decision and signaled it by voice with no limit of time (see Figure 4).

**Figure 3:** Stimulus layout from the eight-alternative forced-choice (8-AFC) task for icons version (left) and toys version (right).

**Figure 4:** Stimulus layout from the assessment task for icons version (left) and toys version (right).

### Data Collection

During the first task, eye-tracking data were obtained using Tobii Studio. It provides the raw data of gaze position in X and Y coordinates according to the stimuli (8-AFC) presented in the screen. A fixation identification algorithm based on the speed of gaze was applied to eye-tracking raw data. The data can be grouped in three classes: (1) if between instants the speed of the gaze was less than a threshold it is considered that a fixation is being made, (2) if it exceeds this speed it is considered as saccade, and (3) and if there has been any error or it is not looking at the screen they are considered non-classified. The identified fixations have been used to model visual attention. Each 8-AFC was segmented in nine areas of interest (AOI) following the 3 × 3 layout: eight AOIs delimited each stimulus (logo or toy) presented, and one delimited the central point used to start the decision-making process. Therefore, each fixation can be assigned to one logo or toy. Using the segmentation, two metrics were computed: total time fixation (TTF), i.e., the summation of the time of all the fixations in one AOI, and visit count (VC), i.e., number of times that the icon or toy was viewed. A visit was defined as the permanency of more than one consecutive fixations in the same AOI, where all of the fixations produce one visit assigned to the AOI. The visit starts when the first fixation starts, and finishes when the last fixation ends, including all the saccades or blinks between the consecutive fixations. Moreover, in order to determine the division between the exploration and the decision-making part of the task, the decision-making instant was defined as the last sample of the last fixation before the visit to the central AOI. All the data processing were perfomed using Matlab R2013.

### Statistical Analysis

The self-assessment in terms of preference of the task 2 was computed to analyze the influence of each dimension in the stimuli: color, character, and eyes/materials. After the descriptive statistics analysis of the design dimensions, linear correlations between preference and visual attention have been performed using Pearson correlations. Moreover, the analysis focused on observing the influence that every dimension had on the children’s gaze behavior. A Kolmogorov-Smirnov normality test was applied to the data used, which showed that the data followed a normal distribution. The statistical method used for the analysis was a multivariable ANOVA (MANOVA) with a Bonferroni correction. Statistical analysis was performed using SPSS 17.0 for Windows™ (IBM SPSS Inc., Chicago, IL, United States).

In addition, we analyze the recognition level of the liking choice of 8-AFC using the visual attention patterns. To this extent, the total fixation time during two sets of visits were analyzed. In particular, the total fixation time of each stimuli AOI in the first four visits were computed to determine if the most viewed icon or toy in the initial exploration can recognize the choice. Alternatively, the total fixation time of each stimuli AOI in the last four visits before the decision-making instant were computed to determine if the most viewed icon or toy in the moments previous to the decision-making can recognize the choice.

Finally, the evolution of the percentage of TTF that each stimulus achieves during the 8-AFC task was analyzed. To this extent, the eight stimuli were characterized in each trial as the choice, i.e., the stimuli that was chosen, and 1–7 distractors, being 1 the (not chosen) stimuli with highest TTF and 7 the one with lowest TTF. During all the instants of a trial, the percentage of TTF that choice and distractors reach was calculated from the start point until this instant. Since the trials do not have the same duration, all of these the trials were synchronized using the instant of the decision-making. The last 3 s of the all icons and toys trials were averaged separately to characterize the time previous to the decision-making moment.

## Results

### Self-Assessment Preferences

The results obtained by the assessment of preference during the second task of the experiment are shown in Figure 5. The results of the 7-point Likert scale can be used for the assessment of the design dimensions used for icons and toys. The children declared the most liked choices of stimulus which were composed among characteristic, color, material, or eye detail.

**Figure 5:** Graphs of results for the assessment of the design dimensions of the icons **(left column)** and toys **(right column)**.

Figure 6 shows linear correlation between preference, TTF, and VC. Icons shows a weak but significant (*p* < 0.05) correlation between preference and TTF (*ρ* = 0.16) and between preference and VC (*ρ* = 0.13). No linear correlations have been found between preference and TTF or VC in toys.

**Figure 6:** Correlations between liking and visual attention. Number in the table shows the Pearson correlation coefficient, and the background is highlighted from red to blue in case of *p* < 0.05. Figure result for icons in left side and figure results for toys in right side.

### Gaze Pattern Differences

Table 1 analyses the independent variable TTF with all the factors [gender, character, color, and eye detail (see Figure 1, left column)] for icons. The gender factor [*F* (9.067), *p* = 0.003] presented a significant main effect (*p* < 0.05). There was no significant interaction between factors. The fixation time (s) differed significantly between boys (mean = 0.546, std = 0.707) and girls (mean = 0.383, std = 0.434). The independent variable VC was also analyzed with all the factors [gender, character, color, and eye detail (see Figure 1, left column)] for icons. There was presented a significant main effect (*p* < 0.05) between factors. Gender*Character interaction [*F* (3.856), *p* = 0.004], Gender*Color [*F* (2.388), *p* = 0.050], Character*Eye detail [*F* (1.902), *p* = 0.018], and Color*Eye detail [*F* (3.708), *p* = 0.000].

**Table 1:** Statistical result of multivariable ANOVA (MANOVA) for independent variables for icons.

Source	*SS*	*dF*	*MS*	*F*	*p*
**Total time fixation**					
Gender	3.529	1	3.529	9.067	0.003^*^
Character	1.561	4	0.390	1.003	0.405
Color	1.375	4	0.344	0.883	0.473
Eye detail	0.930	4	0.233	0.598	0.665
Color*Eye detail	12.429	16	0.777	1.996	0.011^*^
**Visit count**					
Gender*Character	30.573	4	7.643	3.856	0.004^**^
Gender*Color	18.932	4	4.733	2.388	0.050^**^
Gender*Eye details	6.302	4	1.576	0.795	0.529
Character*Color	17.839	16	1.115	0.563	0.912
Character*Eye detail	60.304	16	3.769	1.902	0.018^**^
Color*Eye detail	117.590	16	7.349	3.708	0.000^**^

R Squared = 0.195 (^*^Adjusted R Squared = 0.050). R Squared = 0.226 (^**^Adjusted for R Squared = 0.086).

Table 2 shows the analysis of the independent variable TTF with all the factors [gender, character, color, and material (see Figure 1, right column)] for toys. Material factor [*F* (2.461), *p* = 0.044] presented a significant main effect (*p* < 0.05). There was no significant interaction between factors. The fixation time (seconds) differed significantly between metal (mean = 0.898, std = 1.252), furry (mean = 0.696, std = 1.134), plastic (mean = 0.604, std = 1.090), wood (mean = 0.555, std = 0.827), and cloth (mean = 0.498, std = 0.630). The final analysis was made for the independent variable VC with complete factors [gender, character, color, and material (see Figure 1, right column)] for toys. Gender factor [*F* (2.461), *p* = 0.044] presented a significant main effect (*p* < 0.05). The visit count (times) differed significantly between boys (mean = 2.023, std = 3.14) and girls (mean = 1.491, std = 1.427). There was no significant interaction between factors.

**Table 2:** Statistical result of MANOVA for independent variables for toys.

Source	*SS*	*dF*	*MS*	*F*	*p*
**Total time fixation**					
Gender	2.324	1	2.324	2.182	0.140
Character	8.836	4	2.209	2.074	0.082
Color	2.919	4	0.730	0.685	0.602
Material	10.484	4	2.621	2.461	0.044^*^
**Visit count**					
Gender	34.401	1	34.401	4.414	0.036^**^
Character	22.289	4	5.572	0.715	0.582
Color	46.938	4	11.734	1.506	0.199
Material	20.304	4	5.076	0.651	0.626

R Squared = 0.147 (^*^Adjusted R Squared = 0.017). R Squared = 0.132 (^**^Adjusted for R Squared = 0.000).

### Recognizing the Choice With Visual Attention

Table 3 analyzes the gaze pattern during the four first and four last visits in both icons and toys. The number of visits and the total fixation time of the stimulus (icon and toy) chosen were higher in the last four visits than in the four first visits in both cases. Moreover, the chosen stimulus is the one with the longest fixation time during the last four visits, 67.2% of times for icons and 71.2% for toys. These results are considerably higher than the fixation time computed in the first four visits (23.0 and 15.2%, respectively). In addition, the chosen stimulus is within the top two stimuli with highest fixation time in 82.0 and 84.8% of times for icons and toys, respectively.

**Table 3:** Analysis of the first four and last four dwells in each trial in the 8-AFK task.

Stimulus	Visit set	# of visits to chosen stimulus (ms)	Chosen stimulus total fixation time (ms)	Chosen stimulus is top fixation time (%)	Chosen stimulus within top two fixation time (%)
Icons	First four	0.607 (0.714)	178 (295)	23.0	32.8
	Last four	1.410 (0.761)	906 (678)	67.2	82.0
Toys	First four	0.627 (0.828)	172 (297)	15.2	27.1
	Last four	1.610 (0.891)	1,167 (799)	71.2	84.8

# of visits and total fixation time are shown using mean and standard deviation.

### Analysis of Distractors

Figure 7 shows the proportion of total fixation time during the task that has each stimulus in the last 3 s before the decision-making moment. The data for the version of the icon tasks and toys were plotted separately, collapsing all participants and trials. In both cases, the five stimuli most viewed (the chosen one and the first four distractors) are relatively close 3 s before the decision-making instant. For toys, between 2.5 and 1.5 s before the decision, the future choice and first distractor grow in terms of proportion of TTF. In the last 1.5 s, all distractors decrease, meanwhile, the choice highly increases their TTF overtaking the first distractor. The icons follow the same patterns, but the moment when the choice overtakes the first distractor is 1 s before instead of 1.5.

**Figure 7:** Plots of the proportion of time extracted by chosen stimulus or distractor stimulus by eye-tracking (ranked by total fixation time). Plot result for icons choice and distractor (left) and plot result for toys choice and distractor (right).

## Discussion

The purpose of this research is to analyze the use of visual attention for evaluating children preferences, allowing to evaluate the decision-making processes beyond the classical self-report method. Figure 5 shows the self-assessment preference of each of the stimuli presented and obtained in verbal report of task 2. This assessment helped to understand the implicit perception of design dimensions for icons and toys. The assessment revealed which elements were more liked or less liked by their aesthetic or active elements, including emotional ones (Green-Armytage, 2006; Hertenstein et al., 2013; Helo et al., 2014; Joško-Brakus et al., 2014; Kareklas et al., 2014). However, these evaluations are not capable of knowing to know information beyond the implicit perception of children. Using the information extracted from eye-tracking. A factor analysis was performed where the fixation and visit variables could provide more information about the evaluation, mainly which elements were the most observed or most visited by the children. The first result observed for icons assessment with the TTF variable was the difference between how boys and girls perceiving the icons considering all the design dimensions. Boys on average spent 0.55 s observing the icon, while girls spent only 0.38 s. The second interesting result was how the VC variable on the icons revealed that the gender determines an interaction between design dimensions (color, eye-detail, and character). Boys and girls visit each icon differently depending on the design dimensions. These two results reveal deeper information about the icon assessment. Without having to ask the children which dimensions are the most liked, we can know which is the most observed and which is the most visited in the decision-making process. Also, the other factor analysis was made with the variables of TTF and VC for toys assessment. The first result observed for toys assessment with the TTF variable was the difference between how the material determines the fixation time. Metal is the most viewed, followed by furry and the least seen is the cloth material. The final analysis for this information using the variables extracted from the eye movement was VC. In the toy’s assessment, the gender determined the number of visits that were made by the children. Boys visited a toy 2 times on average, while girls generally visited toys only 1.5 times on average. These two results reveal information that supports how the children were able to determine their choice of which toys were most liked. The material was a design dimension that caught their attention (Kwon et al., 2002; Lin, 2010; Festila and Chrysochou, 2018) and how boys need to visit more times than girls to do a decision-making. The results obtained using the traditional methods of icons and toys assessment were enhanced with the use of the data extracted from eye movement. This shows how the use of implicit measures can give deeper insights of the elements that were the determining factors in decision-making, as well as show the differences in behavior that a sample of people can have, in this study, gender was a determining factor.

In the present study, the method to recognition of decision-making with eye movement contribute beyond self-report was further explored. The 8-AFC task (Glaholt et al., 2009; Glaholt and Reingold, 2012) was using in multi-stimuli arrays for understanding the effect of eye movements and selection during preference process for children behavior. This task provided information on children’s gaze behavior, providing additional insights that those already extracted in the analysis above. The information extracted from the two variables of eye movement and the design dimensions assessment were the base of this study. We explore the recognition level of the liking choice of 8-AFC using the visual attention patterns. To this propose, two sets of time-windows were analyzed: the first four visits and the last four visits. The results show that the first four visits were not able to recognize the future choice of the children, achieving 23.0 and 15.2% in icons and toys, respectively. Therefore, the results indicate that the preference for an item of the children is not correlated with the visual attention on the first seconds of exploration. On the other hand, the TTF of the last four visits allow to recognize the choice of a participant in 67.2 and 71.2% of the cases, which is considerably higher that the chance level in an 8-class problem (chance = 12.5%), assuming that the stimuli with higher TTF in this time-windows is the chosen one. Moreover, the final choice is taken from the top two stimuli with higher TTF in the 82.0 and 84.8% (in icons and toys, respectively) of times during the last four visits, in contrast to 32.8 and 84.8% when the first four visits are analyzed. Table 3 shows the VC and TTF metrics of the chosen stimulus, where the values are always higher in the last four visits than in the first four for both icons and toys. The evolution of the percentage of TTF that each stimulus reaches during the 8-AFC task was also analyzed to characterize the choice dynamics and a decision is made in children’s visual attention. Figure 7 shows, in a graphic representation, the choice and the first four distractors in timeline of 3 s before the instant when the decision is made. Between 2.5 and 1.5 s before a decision is made, the choice and first distractor increase their accumulated TTF. The second distractor also appears but smoothly. In the case of icons, this phase was finalized 1 s before the decision. This suggests that, within these time windows, the subject is evaluating between 2 and 3 choices. Finally, from this point of view, the accumulated TTF of choice overtakes the first distractor, and it in this time window where the decision is matured. This process takes 1 s for icons and 1.5 s for toys. It suggests that the decision-making process regarding toys takes more time, probably derived from the fact that toys are more complex stimuli and need more mental effort. This time can be used as an implicit measure of the effort needed to make a decision, and can help future designers, complementing classical self-reports.

The findings of this paper open possibilities to combine traditional self-report and eye movement techniques contribute with techniques that dive beyond self-report, and how this method reveal relevant information of people’s behavior. The results of the first task of the experiment show similar results in the selection of the preference among different distractors (Shimojo et al., 2003; Simion and Shimojo, 2006, 2007; Glaholt and Reingold, 2009, 2012) and repeats the findings of Glaholt and Reingold (2012) and Mitsura and Glaholt (2014), where chosen stimuli dynamics can become an automatic recognition model using children eye movements. The result show of the second tasks show the analysis complexity that the assessment of the design dimensions stimuli can represent, this was addressed in a way such that the aesthetic implications or attributes such as color, material, or textures (Kwon et al., 2002; Green-Armytage, 2006; Lin, 2010; Hertenstein et al., 2013; Helo et al., 2014; Joško-Brakus et al., 2014; Kareklas et al., 2014; Festila and Chrysochou, 2018) could be observed through the fixation and visits.

However, it is still possible to go deeper into studies that focus on determining the relevance of each of these elements in decision-making and the heuristic recognition theory. The assessment results of icons and toys preference feed the information described by Pachur et al. (2011) on familiarity and inference in decision-making. Also, the main idea of this paper was to use simple stimuli that children could make quick and simple choice, following the notion presented by Marewski et al. (2009) and Arkes et al. (2016) for the consistency and simplicity in cognitive process. Finally, this type of paper contribution helps to understand human behavior and regardless of certain restrictions that a self-report may have in research of this nature (Song et al., 1994; Chambers, 2002; Sturgess et al., 2002; Kuijpers et al., 2014), we can continue to create relationships with adjacent theories and methods.

## Conclusions

The current paper gives a relevant empirical result of a method that contributes to a better knowledge of the decision-making process in children, providing an interesting technique that goes beyond self-reports. Compared to other methods that use neuroscience tools, this one has a low complexity of implementation and good accessibility due to the type of technology that is required. Furthermore, this paper presents the implementation of our method with a sample of subjects, specifically children, who pose different challenges in order to analyze their behavior. As highlighted in several previous works, the use of eye-tracking can help to have an implicit measurement that can be used as an alternative or a complement to the collection of traditional data based on explicit measures by self-reporting or questionnaires. Future studies are planned to work with a bigger sample size, and other age segments, to confirm the results obtained in the present work.

## Data Availability Statement

The datasets presented in this article are not readily available because this experiement has a raw data and process in Matlab and SPSS data base. Requests to access the datasets should be directed to jcrojasl@tec.mx.

## Ethics Statement

The studies involving human participants were reviewed and approved by Universitat Politecnica de Valencia. Written informed consent to participate in this study was provided by the participants’ legal guardian/next of kin.

## Author Contributions

All authors have contributed to the manuscript as follows: J-CR designed the study and supervised the whole study. JM-M conducted the eye-tracking raw data. J-CR and MC conducted the statistical analyses. J-CR, JM-M, and JMAA wrote the original manuscript. MC revised the manuscript. All authors assisted in the revision process, read, and approved the final manuscript.

### Conflict of Interest

This study was part of the realization of the doctoral thesis of one of the authors. The authors declare that the research was conducted in the absence of any commercial or financial relationships that could be construed as a potential conflict of interest.

## References

[ref1] ArkesH.GigerenzerG.HertwigR. (2016). How bad is incoherence? Decision 3, 20–39. 10.1037/dec0000043

[ref2] BellL.VogtJ.WillemseC.RoutledgeT.ButlerL. T.SakakiM. (2018). Beyond self-report: a review of physiological and neuroscientific methods to investigate consumer behavior. Front. Psychol. 9:1655. 10.3389/fpsyg.2018.01655, PMID: 30245657PMC6137131

[ref3] BlancoS.DietmannS.FloresJ. V.HussainS.KutterC.HumphreysP.. (2014). Aberrant methylation of tRNAs links cellular stress to neuro-developmental disorders. EMBO J. 33, 2020–2039. 10.15252/embj.201489282, PMID: 25063673PMC4195770

[ref4] ChambersC. (2002). Developmental differences in children’s use of rating scales. J. Pediatr. Psychol. 27, 27–36. 10.1093/jpepsy/27.1.27, PMID: 11726677

[ref5] ChoE.KimY. K. (2012). The effects of website designs, self-congruity, and flow on behavioral intention. Int. J. Des. 6, 31–41.

[ref6] CowartK. O.FoxG. L.WilsonA. E. (2008). A structural look at consumer innovativeness and self-congruence in new product purchases. Psychol. Mark. 25, 1111–1130. 10.1002/mar.20256

[ref7] CroneE. A.RidderinkhofK. R. (2011). The developing brain: from theory to neuroimaging and back. Dev. Cogn. Neurosci. 1, 101–109. 10.1016/j.dcn.2010.12.001, PMID: 22436435PMC6987573

[ref8] DjamasbiS.SiegelM.TullisT. (2010). Generation Y, web design, and eye tracking. Int. J. Hum. Comput. Stud. 68, 307–323. 10.1016/j.ijhcs.2009.12.006

[ref9] FantzR. L. (1963). Pattern vision in newborn infants. Science 140, 296–297. 10.1126/science.140.3564.296, PMID: 17788054

[ref10] FantzR. L. (1964). Visual experience in infants: decreased attention to familiar patterns relative to novel ones. Science 146, 668–670. 10.1126/science.146.3644.668, PMID: 14191712

[ref11] FestilaA.ChrysochouP. (2018). Implicit communication of food product healthfulness through package design: a content analysis. J. Consum. Behav. 17, 461–476. 10.1002/cb.1732

[ref12] GigerenzerG.GoldsteinD. G. (2011). The recognition heuristic: a decade of research. Judgm. Decis. Mak. 6, 100–121.

[ref13] GlaholtM. G.ReingoldE. M. (2009). The time course of gaze bias in visual decision tasks. Vis. Cogn. 17, 1228–1243. 10.1080/13506280802362962

[ref14] GlaholtM. G.ReingoldE. M. (2012). Direct control of fixation times in scene viewing: evidence from analysis of the distribution of first fixation duration. Vis. Cogn. 20, 605–626. 10.1080/13506285.2012.666295

[ref15] GlaholtM. G.WuM. -C.ReingoldE. M. (2009). Predicting preference from fixations. PsychNology J. 7, 141–158. 10.1037/e527342012-455

[ref16] Green-ArmytageP. (2006). The value of knowledge for colour design. Color Res. Appl. 31, 253–269. 10.1002/col.20222

[ref400] GrunertK. G.BredahlL.BrunsøK. (2004). Consumer perception of meat quality and implications for product development in the meat sector—a review. Meat Science. Meat Sci. 66, 259–272. 10.1016/s0309-1740(03)00130-x22064127

[ref17] HeljakkaK.IhamäkiP. (2019). “Toys that mobilize: past, present and future of phygital playful technology.” Advances in Intelligent Systems and Computing. 625–640.

[ref300] HeloA.PannaschS.SirriL.RämäP. (2014). The maturation of eye movement behavior: scene viewing characteristics in children and adults. Vis. Res. 103, 83–91. 10.1016/j.visres.2014.08.00625152319

[ref18] HertensteinJ. H.PlattM. B.VeryzerR. W. (2013). What is “Good Design”?: an investigation of the complexity and structure of design. Design Manag. J. 8, 8–21. 10.1111/dmj.12000

[ref19] HsuM. (2017). Neuromarketing: inside the mind of the consumer. Calif. Manag. Rev. 59, 5–22. 10.1177/0008125617720208

[ref20] HsuM.YoonC. (2015). The neuroscience of consumer choice. Curr. Opin. Behav. Sci. 5, 116–121. 10.1016/j.cobeha.2015.09.005, PMID: 26665152PMC4671287

[ref21] HubertM. (2010). Does neuroeconomics give new impetus to economic and consumer research? J. Econ. Psychol. 31, 812–817. 10.1016/j.joep.2010.03.009

[ref22] HubertM.KenningP. (2008). A current overview of consumer neuroscience. J. Consum. Behav. 7, 272–292. 10.1002/cb.251

[ref23] HultG. T. M.SharmaP. N.MorgesonF. V.3rdZhangY. (2019). Antecedents and consequences of customer satisfaction: do they differ across online and offline purchases? J. Retail. 95, 10–23. 10.1016/j.jretai.2018.10.003

[ref24] Joško-BrakusJ.SchmittB. H.ZhangS. (2014). Experiential product attributes and preferences for new products: the role of processing fluency. J. Bus. Res. 67, 2291–2298. 10.1016/j.jbusres.2014.06.017

[ref25] KareklasI.BrunelF. F.CoulterR. A. (2014). Judgment is not color blind: the impact of automatic color preference on product and advertising preferences. J. Consum. Psychol. 24, 87–95. 10.1016/j.jcps.2013.09.005

[ref26] KarmarkarU. R.PlassmannH. (2017). Consumer neuroscience: past, present, and future. Organ. Res. Methods 22, 174–195. 10.1177/1094428117730598

[ref27] KuijpersR.OttenR.VermulstA.EngelsR. (2014). Reliability and construct validity of a child self-report instrument. Eur. J. Psychol. Assess. 30, 40–47. 10.1027/1015-5759/a000166

[ref28] KwonO. B.KimC. R.LeeE. J. (2002). Impact of website information design factors on consumer ratings of web-based auction sites. Behav. Inform. Technol. 21, 387–402. 10.1080/0144929021000050256

[ref500] LaforetS. (2011). Brand names on packaging and their impact on purchase preference. J. Cust. Behav. 10, 18–30. 10.1002/cb.343, PMID: 14191712

[ref29] LăzăroiuG.PeraA.Ștefănescu-MihăilăR. O.MircicăN.NegurităO. (2017). Can neuroscience assist us in constructing better patterns of economic decision-making? Front. Behav. Neurosci. 11:188. 10.3389/fnbeh.2017.00188, PMID: 29066963PMC5641305

[ref30] LiaoH. -I.ShimojoS.YehS. -L. (2013). Happy faces are preferred regardless of familiarity-sad faces are preferred only when familiar. Emotion 13, 391–396. 10.1037/a0030861, PMID: 23356560

[ref31] LiaoH. -I.YehS. -L.ShimojoS. (2011). Novelty vs. familiarity principles in preference decisions: task-context of past experience matters. Front. Psychol. 2:43. 10.3389/fpsyg.2011.00043, PMID: 21713246PMC3110941

[ref32] LiebermanM. D. (2007). Social cognitive neuroscience: a review of core processes. Annu. Rev. Psychol. 58, 259–289. 10.1146/annurev.psych.58.110405.085654, PMID: 17002553

[ref33] LinL. Y. (2010). The relationship of consumer personality trait, brand personality and brand loyalty: an empirical study of toys and video games buyers. J. Prod. Brand Manag. 19, 4–17. 10.1108/10610421011018347

[ref34] LuoM. R. (2006). Applying colour science in colour design. Opt. Laser Technol. 38, 392–398. 10.1016/j.optlastec.2005.06.025

[ref35] MarewskiJ.GaissmaierW.GigerenzerG. (2009). Good judgments do not require complex cognition. Cogn. Process. 11, 103–121. 10.1007/s10339-009-0337-0, PMID: 19784854PMC2860098

[ref36] MitsuraT.GlaholtM. G. (2014). Gaze bias during visual preference judgements: effects of stimulus category and decision instructions. Vis. Cogn. 22, 11–29. 10.1080/13506285.2014.881447

[ref37] MoriiM.SakagamiT. (2015). The effect of gaze-contingent stimulus elimination on preference judgments. Front. Psychol. 6:1351. 10.3389/fpsyg.2015.01351, PMID: 26441727PMC4563161

[ref38] OchsnerK.GrossJ. (2005). The cognitive control of emotion. Trends Cogn. Sci. 9, 242–249. 10.1016/j.tics.2005.03.010, PMID: 15866151

[ref39] PachurT.ToddP.GigerenzerG.SchoolerL.GoldsteinD. (2011). The recognition heuristic: a review of theory and tests. Front. Psychol. 2:147. 10.3389/fpsyg.2011.00147, PMID: 21779266PMC3132682

[ref40] ParkJ.ShimojoE.ShimojoS. (2010). Roles of familiarity and novelty in visual preference judgments are segregated across object categories. Proc. Natl. Acad. Sci. U. S. A. 107, 14552–14555. 10.1073/pnas.1004374107, PMID: 20679235PMC2930416

[ref41] PoelsK.DewitteS. (2006). How to capture the heart? Reviewing 20 years of emotion measurement in advertising. J. Advert. Res. 46, 18–37. 10.2501/S0021849906060041

[ref42] QuQ.GouF. (2019). Can eye movements be effectively measured to assess product design?: gender differences should be considered. Int. J. Ind. Ergon. 72, 281–289. 10.1016/j.ergon.2019.06.006

[ref43] RojasJ. -C.ConteroM.BartomeuN.GuixelesJ. (2015). Using combined bipolar semantic scales and eye tracking metrics to compare consumer perception of real and virtual bottles. Packag. Technol. Sci. 28, 1047–1056. 10.1002/pts.2178

[ref44] SaegusaC.IntoyJ.ShimojoS. (2015). Visual attractiveness is leaky: the asymmetrical relationship between face and hair. Front. Psychol. 6:377. 10.3389/fpsyg.2015.00377, PMID: 25914656PMC4390982

[ref45] ShimojoS.SimionC.ShimojoE.ScheierC. (2003). Gaze bias both reflects and influences preference. Nat. Neurosci. 6, 1317–1322. 10.1038/nn1150, PMID: 14608360

[ref46] SimionC.ShimojoS. (2006). Early interactions between orienting, visual sampling and decision making in facial preference. Vis. Res. 46, 3331–3335. 10.1016/j.visres.2006.04.019, PMID: 16765404

[ref47] SimionC.ShimojoS. (2007). Interrupting the cascade: orienting contributes to decision making even in the absence of visual stimulation. Percept. Psychophys. 69, 591–595. 10.3758/bf03193916, PMID: 17727112

[ref48] SmidtsA.HsuM.SanfeyA. G.BoksemM. A.EbsteinR. B.HuettelS. A. (2014). Advancing consumer neuroscience. Mark. Lett. 25, 257–267. 10.1007/s11002-014-9306-1

[ref49] SolnaisC.Andreu-PerezJ.Sánchez-FernándezJ.Andréu-AbelaJ. (2013). The contribution of neuroscience to consumer research: a conceptual framework and empirical review. J. Econ. Psychol. 36, 68–81. 10.1016/j.joep.2013.02.011

[ref50] SongL.SinghJ.SingerM. (1994). The youth self-report inventory: a study of its measurements fidelity. Psychol. Assess. 6, 236–245. 10.1037/1040-3590.6.3.236

[ref51] StantonS. J.Sinnott-ArmstrongW.HuettelS. A. (2017). Neuromarketing: ethical implications of its use and potential misuse. J. Bus. Ethics 144, 799811. 10.1007/s10551-016-3059-0

[ref52] SteinhauserJ.JanssenM.HammU. (2019). Consumers’ purchase decisions for products with nutrition and health claims: what role do product category and gaze duration on claims play? Appetite 141:104337. 10.1016/j.appet.2019.104337, PMID: 31260708

[ref53] SturgessJ.RodgerS.OzanneA. (2002). A review of the use of self-report assessment with young children. Br. J. Occup. Ther. 65, 108–116. 10.1177/030802260206500302

[ref54] TanakaJ.WeiskopfD.WilliamsP. (2001). The role of color in high-level vision. Trends Cogn. Sci. 5, 211–215. 10.1016/s1364-6613(00)01626-0, PMID: 11323266

[ref55] Van der LaanL. N.HoogeI. T. C.De RidderD. T. D.ViergeverM. A.SmeetsP. A. M. (2015). Do you like what you see? The role of first fixation and total fixation duration in consumer choice. Food Qual. Prefer. 39, 46–55. 10.1016/j.foodqual.2014.06.015

[ref56] WangY. J.MinorM. S. (2008). Validity, reliability, and applicability of psychophysiological techniques in marketing research. Psychol. Mark. 25, 197–232. 10.1002/mar.20206

[ref57] WedelM.PietersR. (2006). Eye tracking for visual marketing. Found. Trends Mark. 1, 231–320. 10.1561/1700000011

[ref58] YaramothuC.SantosE. M.AlvarezT. L. (2018). Effects of visual distractors on vergence eye movements. J. Vis. 18:2. 10.1167/18.6.2, PMID: 30029212PMC5987826

